# CircRNA circPDSS1 promotes bladder cancer by down-regulating miR-16

**DOI:** 10.1042/BSR20191961

**Published:** 2020-01-07

**Authors:** Qinnan Yu, Pei Liu, Guangye Han, Xiangdong Xue, Derong Ma

**Affiliations:** 1 Department of Urology, The First Affiliated Hospital of Xinxiang Medical College, Weihui City, Henan Province 453100, P.R. China; 2 Department of Urology, Gansu Provincial People’s Hospital, Lanzhou City 730000, Gansu Province, P.R. China

**Keywords:** circPDSS1, miR-16, urothelial bladder cancer

## Abstract

**Background:** Circular RNA (circRNA) circPDSS1 is a recently identified oncogene in gastric cancer, while its roles in other types of cancer are unknown. We investigated the functions of circPDSS1 in urothelial bladder cancer (UBC).

**Materials and methods:** Seventy-two patients (50 males and 22 females, age 38–69 years, mean: 52.3 ± 6.3 years) with UBC were enrolled in Gansu Provincial People’s Hospital from August 2015 to August 2018. RT-qPCR was used to measure gene expression levels in both biopsies from UBC patients and *in vitro* cultivated HT-1197 and UMUC3 cells. Cell transfections were performed to analyze gene interactions. Cell proliferation, transwell migration and invasion assays were performed to analyze the effects of transfections on HT-1197 and UMUC3 cell proliferation, migration and invasion, respectively.

**Results:** We found that circPDSS1 was up-regulated in UBC. Expression levels of circPDSS1 were increased with increase in clinical stages. MiR-16 was down-regulated and correlated with circPDSS1 in UBC. Overexpression of circPDSS1 led to down-regulation of miR-16, while miR-16 overexpression failed to significantly affect circPDSS1. Overexpression of circPDSS1 led to increased proliferation, invasion and migration rates of UBC cells. Overexpression of miR-16 not only led to inhibited proliferation, invasion and migration of UBC cells, but also attenuated the effects of circPDSS1 overexpression.

**Conclusion:** Therefore, circRNA circPDSS1 may promote UBC by down-regulating miR-16.

## Introduction

Bladder cancer is the second most commonly diagnosed malignancy developing from urologic system [1]. In 2013, bladder cancer affected approximately 70000 new cases and caused more than 15000 deaths in the United States [2]. Noninvasive urothelial carcinoma accounts for 70% of all bladder tumors, and the rest are muscle-invasive diseases [3]. Radical cystectomy is the most common treatment strategy for muscle-invasive tumors, while prognosis is usually poor even after active treatment. [4] At present, the 5-year survival of muscle-invasive bladder cancer patients remains below 60% [4]. Therefore, novel therapeutic targets are always needed to improve the treatment outcomes of bladder cancer patients.

Circular RNAs (circRNAs) are RNA molecules, unlike linear RNAs, with 3′- and 5′-ends covalently joined to form closed continuous loops [5]. To date, more than 2000 different circRNA species in human have been identified, while the function of most circRNAs remains unclear [6,7]. It is known that circRNAs are critical determinants in cancer biology [8,9], and certain circRNAs may serve as biomarkers for cancer diagnosis and prognosis [10]. CircRNA circPDSS1 is a recently identified oncogenic RNA in gastric cancer [11], while its roles in other types of cancer are unknown. Our study was thus carried out to investigate the role of circPDSS1 in urothelial bladder cancer (UBC), which is the most common subtype of bladder cancer. We also explored the potential interactions between circPDSS1 and with miR-16, which inhibits bladder cancer [12].

## Materials and methods

### Research subjects

Our study included 72 patients (50 males and 22 females, age 38–69 years, mean: 52.3 ± 6.3 years) with UBC in Gansu Provincial People’s Hospital from August 2015 to August 2018. UBC was confirmed by pathological test. Inclusion criteria: (1) UBC patients who were treated for the first time; (2) patients signed informed consent. Exclusion criteria: (1) patients complicated with other diseases; (2) patients who were transferred from other hospitals or treatment had been performed before admission. According to AJCC staging, there were 16 cases at stage I, 18 at stage II, 22 at stage III and 16 at stage IV. Ethics Committee of Gansu Provincial People’s Hospital approved the present study before the admission of patients. Experiments using human materials were performed in strict accordance with Declaration of Helsinki.

### Specimens and cell lines

Specimens of tumor and adjacent (2 cm around tumors) healthy tissues were collected from each patient through biopsy. Our study included HT-1197 and UMUC3 two human bladder cancer cell lines (ATCC, U.S.A.). Eagle’s Minimum Essential Medium containing 10% fetal bovine serum (FBS) was used as cell culture medium, and cell culture conditions were 37°C and 5% CO_2_.

### Total RNA extractions and RT-qPCR

To detect the expression of circPDSS1, total RNAs were extracted from tissue specimens and *in vitro* cultivated cell using RNAzol reagent (Sigma–Aldrich, St. Louis, MO, U.S.A.). SuperScript IV Reverse Transcriptase (Thermo Fisher Scientific) and Applied Biosystems™ Power™ SYBR™ Green Master Mix were used to perform reverse transcriptions and prepare PCR mixtures, respectively. To detect the expression of miR-16, miRNeasy Mini Kit (QIAGEN) was used to extract miRNAs, miScript II RT Kit (QIAGEN) was used to perform microRNA reverse transcription and miScript SYBR® Green PCR Kit (QIAGEN) was used to prepare PCR mixtures. PCRs were performed with GAPDH as the endogenous control of circPDSS1 and U6 as the endogenous control of miR-16. Primer sequences were: 5′-GTGGTGCATGAGATCGCCT-2′ (forward) and 5′-GGGTTGTGTGATGAAACCTG-3′ for CircPDSS1; 5′-GAAGGTGAAGGTCGGAGTCGAPD-2′ (forward) and 5′-GAAGATGGTGATGGGATTT-3′ for GAPDH; 5′-TAGCAGCACGTAAATATTGGCG-3′ (forward) for miR-16. Reverse primer and U6 primers were included in the kit. PCR products were sequenced to ensure correct products were obtained. Primers of CircPDSS1 were on the different sides of the ligation site to ensure the specific amplification of circRNA. No-template reactions were used as negative control (NC) reactions. All data normalization were performed based on 2^−ΔΔ*C*_T_^ method.

### Cell transfection

PcDNA3.1 vector expressing circPDSS1 (circ_0093398, circBase) was constructed by Sangon (Shanghai, China). MiR-16 mimic and scrambled NC miRNA were purchased from Sigma–Aldrich. Cells of HT-1197 and UMUC3 cell lines were cultivated at 37°C in a 5% CO_2_ incubator to reach 70–80% confluence, and cell transfections were performed using Lipofectamine 2000 (Invitrogen, Carlsbad, U.S.A.). The doses of vectors and miRNAs were 10 and 40 nM, respectively. The ratio of Lipofectamine™ 2000 (in µl):DNA (in µg) was 3:1. Un-transfected cells and cells transfected with empty vectors were used as control and NC, respectively. Cells were harvested at 24 h after transfection for subsequent experiments.

### Cell proliferation assay

In the present study, cell proliferation abilities were tested through *in vitro* cell proliferation assay using Cell Counting Kit-8 kit (ab228554, Abcam) at 24 h after transfection. Single cell suspensions (5 × 10^4^ cells/ml) were prepared using Eagle’s Minimum Essential Medium (10% FBS). Cell suspensions were cultivated in a 96-well plate (0.1 ml per well) 37°C in a 5% CO_2_ incubator. CCK-8 solution (10 μl) was added every 24 h until 96 h. Cells were then cultivated for further 4 h and 10 μl DMSO was added. Finally, OD values (450 nm) were measured to represent cell proliferation ability. For data normalization, OD values of control group at 96 h were set to ‘100’, and all other time points and other groups were normalized to control group.

### Transwell migration and invasion assay

In the present study, cell invasion and migration abilities were tested through Transwell assays at 24 h after transfection. Single cell suspensions (5 × 10^4^ cells/ml) were prepared using serum-free Eagle’s Minimum Essential Medium. Cell suspension was added into the upper chamber (0.1 ml per well), while the lower chamber was filled with Eagle’s Minimum Essential Medium (20% FBS). Cells were cultivated for 3 h, followed by upper chamber membrane staining for 20 min using 0.5% Crystal Violet (Sigma–Aldrich, U.S.A.) at 25°C. Stained cells were observed under an optical microscope. Before invasion assay, Matrigel (356234, Millipore, U.S.A.) was used to pre-coat the upper chamber at room temperature for 12 h. The number of invading or migrating cells of control group was set to ‘100’, and all other groups were normalized to control group.

### Statistical analysis

Three biological replicates were performed for each experiment, and mean ± standard deviation was used to express all data. Comparisons between two types of tissues were performed by paired *t* test. Comparisons among different clinical stages and among different cell treatment groups were performed by ANOVA (one-way) and Tukey’s test. Linear regression was performed to investigate the correlations between expression levels of circPDSS1 and miR-16. Differences with *P*<0.05 were considered to be statistically significant.

## Results

### CircPDSS1 was up-regulated in UBC tissues and affected by clinical stages

To detect the differential expression of circPDSS1, RT-qPCR was performed to measure the expression levels of circPDSS1 in both tumor and adjacent healthy tissues (normal tissues) of UBC patients. It was observed that circPDSS1 was significantly up-regulated in cancer tissues compared with normal tissues (Figure 1A, *P*<0.05). In addition, significant increases in expression levels of circPDSS1 in tumor tissues were found with the increase in clinical stages (Figure 1B, *P*<0.05).

**Figure 1:** circPDSS1 was up-regulated in UBC tissues and affected by clinical stages RT-qPCR was performed to measure the levels of circPDSS1 expression in both cancer tissues and adjacent healthy tissues (**A**). PCRs were performed in triplicate manner and mean values were presented and compared by paired *t* test. Differences in expression levels of circPDSS1 in tumor tissues among patients with different clinical stages were analyzed by ANOVA (one-way) combined with Tukey’s test (*, *P*<0.05).

### MiR-16 was down-regulated in cancer tissues and was inversely correlated with circPDSS1

RT-qPCR experiment was also performed to measure the expression levels of miR-16. Different from the expression pattern of circPDSS1, miR-16 was significantly down-regulated in tumor tissues compared with normal tissues of UBC patients (Figure 2A, *P*<0.05). Linear regression was performed to investigate the correlations between expression levels of circPDSS1 and miR-16. Interestingly, expression levels of miR-16 were significantly and inversely correlation with expression levels of circPDSS1 only in tumor tissues (Figure 2B), but not in adjacent healthy tissues (Figure 2C).

**Figure 2:** MiR-16 was down-regulated in cancer tissues and was inversely correlated with circPDSS1 Expression levels of miR-16 in tumor tissues and normal tissues of UBC patients were also measured by RT-qPCR (**A**). PCRs were performed in triplicate manner and mean values were presented and compared by paired *t* test. Linear regression was performed to investigate the correlations between expression levels of circPDSS1 and miR-16 across tumor tissues (**B**) and adjacent healthy tissues (**C**), (*, *P*<0.05).

### CircPDSS1 is a negative upstream regulator of miR-16 in bladder cancer cells

To further explore the interactions between circPDSS1 and miR-16, circPDSS1 and miR-16 were expressed in cells of both HT-1197 and UMUC3 cell lines. For HT-1197 cell line, comparing with control (C) and NC groups, overexpression of circPDSS1 led to down-regulation of miR-16 (*P*<0.05), while miR-16 overexpression failed to significantly affect circPDSS1 expression (Figure 3A). Similar results were observed in UMUC3 cell line (Figure 3B).

**Figure 3:** circPDSS1 is a negative upstream regulator of miR-16 in bladder cancer cells HT-1197 (**A**) and UMUC3 (**B**) cells were transfected with circPDSS1 expression vector or miR-16 mimic. Overexpression of circPDSS1 and miR-16 was confirmed by RT-qPCR. The effects of circPDSS1 overexpression on miR-16 and the effects of miR-16 overexpression on circPDSS1 were also analyzed by RT-qPCR. All experiments were repeated three times and mean values were presented and compared (*, *P*<0.05).

### CircPDSS1 overexpression regulated UBC cell behaviors

Compared with NC and control (C) groups, significantly increased proliferation (Figure 4), migration (Figure 5A) and invasion (Figure 5B) rates were observed after the overexpression of circPDSS1 (*P*<0.05). In contrast, overexpression of miR-16 led to inhibited proliferation, migration and invasion of cancer cells (*P*<0.05). In addition, overexpression of miR-16 also attenuated the effects of circPDSS1 overexpression (*P*<0.05). Therefore, in the regulation of UBC behaviors miR-16 is at the downstream of circPDSS1.

**Figure 4:** circPDSS1 overexpression regulated UBC cell behaviors Cell proliferation assay was performed to analyze the effects of circPDSS1 l and miR-16 overexpression on the proliferation of HT-1197 and UMUC3 cells. All experiments were repeated three times and mean values were presented and compared (*, *P*<0.05).

**Figure 5:** circPDSS1 overexpression promoted bladder cancer cell migration and invasion through miR-16 Transwell assays were performed to analyze the effects of circPDSS1 l and miR-16 overexpression on the migration (**A**) and invasion (**B**) of cells of both HT-1197 and UMUC3 cells. All experiments were repeated three times and mean values were presented and compared (*, *P*<0.05).

## Discussion

Function of most circRNAs remains unclear. We found that circPDSS1 was up-regulated in UBC tissues, and circPDSS1 may promote the development of UBC by regulating the behaviors of cancer cells through the down-regulation of tumor suppression miR-16.

The development and progression of UBC requires the involvement of multiple internal and external factors [13]. In spite of the unknown functionality of most circRNAs, a considerable number of studies have shown that dysregulated circRNAs contribute to the pathogenesis pathway of UBC [14,15]. CircRNA MYLK was overexpressed in UBC tissues, and overexpression of MYLK led to promoted cancer progression through the regulation of VEGFA/VEGFR2 signaling pathway [14]. In contrast, circRNA circ-ITCH was down-regulated in UBC, and overexpression of circ-ITCH mediated the inhibition of bladder cancer through the interactions with multiple miRNAs and p21 signaling pathway [15]. circPDSS1 is a recently identified circRNA promotes in gastric cancer [11]. Our study first reported the up-regulated expression of circPDSS1, and our experimental data showed that circPDSS1 played a role as oncogene in UBC by regulating cancer cell behaviors.

MiR-16 is a well-characterized tumor suppressive microRNA in different types of cancer [16,17]. In a recent study, Jiang et al. [12] showed that miR-16 targeted Cyclin D1 to inhibit the development of UBC. Our findings also showed that miR-16 was down-regulated in UBC and overexpression of miR-16 led to inhibited proliferation, migration and invasion of cancer cells. Our study further confirmed the tumor suppressive effects of miR-16 in UBC. It has been reported that miR-16 may interact with certain circRNAs to participate in cancer biology [18]. Interestingly, our study showed that circPDSS1 was likely an upstream inhibitor of miR-16 in UBC. However, no significant correlations between the expression level of circPDSS1 and miR-16 were observed in normal tissues. Our preliminary luciferase reporter assay data also suggest indirect interaction between circPDSS1 and miR-16 (data not shown). Therefore, the interaction between circPDSS1 and miR-16 may be UBC-specific or disease-specific.

In conclusion, circPDSS1 was up-regulated in UBC and may play a role as oncogene in this disease by serving as an upstream inhibitor of tumor suppressor miR-16.

## Abbreviations

AJCC: American Joint Committee on Cancer
circ-ITCH: circular RNA Itchy E3 ubiquitin protein ligase
circRNA: circular RNA
FBS: fetal bovine serum
GAPDH: glyceraldehyde-3-phosphate dehydrogenase
MYLK: myosin light chain kinase
NC: negative control
OD: optical density
RT-qPCR: Quantitative reverse transcription PCR
UBC: urothelial bladder cancer
VEGFA/VEGFR2: vascular endothelial growth factor A/Vascular endothelial growth factor receptor 2
